The article "Application Effect of Silver-Containing Dressings in the Repair of Chronic Refractory Wounds" was published in 2022. Journal: Evid Based Complement Alternat Med.

# Application Effect of Silver-Containing Dressings in the Repair of Chronic Refractory Wounds

**DOI:** 10.1155/2022/3616923

**Published:** 2022-09-10

**Authors:** Rui Wang, Yuan Guo, Bao Li, Jingjing Zheng, Zhishui Tang, Maoguo Shu

**Affiliations:** The First Affiliated Hospital of XI'AN Jiaotong University Plastic and Cosmetic Maxillofacial Surgery, Xi'an, Shanxi 710061, China

## Abstract

Chronic refractory wounds have complicated pathogenesis, repeatedly prolonged course of disease, high difficulty in cure, and may even endanger life due to the spread of wound infection. Silver ion dressing is a new type of dressing applied clinically in recent years. It can prevent infection and promote wound healing by releasing a low level of active silver ions into wound fluid or secretion. Some scholars have found that silver ion dressings can promote the healing of refractory wounds. In this study, 80 cases of chronic refractory wounds treated in our department from June 2019 to January 2022 were selected as the research subjects and the effect of silver ion dressing coverage on the repair of chronic refractory wounds after debridement was explored.

## 1. Introduction

Clinically, wounds are usually divided into acute wounds and chronic wounds according to the time of healing. Acute wounds refer to wounds that can heal spontaneously within 2 weeks. However, due to some adverse factors such as infection, foreign body, and ischemia that affect the wound healing and partially or completely stop the wound healing, the wound that still cannot heal after more than two weeks is clinically called a chronic refractory wound [1, 2]. Chronic refractory wounds (wounds) are common in pressure ulcers, diabetic foot ulcers, venous ulcers, residual burn wounds, traumatic ulcers, vascular extravasation of strongly irritating drugs, and malignant radiation ulcers [3, 4]. These chronically infected wounds have a high probability of clinical infection, which reduces the quality of life of patients and affects the life and health of patients. Moreover, chronic refractory wounds are difficult to manage and often require multiple methods of coordinated intervention, posing great challenges for clinical health care workers [5, 6]. The challenge of how to reduce wound exudation, reduce pain during wound dressing change, and promote wound healing is an urgent problem to be solved by medical staff.

Silver-containing dressings is a new type of dressing used clinically in recent years, which is mainly composed of sodium carboxymethyl fibers and silver. It prevents infection by releasing a low level of active silver ions into wound fluid or secretions and has the effects of absorbing wound exudate and potent sterilization, improving the wound microenvironment while controlling infection, facilitating wound healing recovery, and promoting wound granulation formation [7, 8]. However, there are still few reports on its clinical application effects and mechanism in China. Based on this, the aim of this study was to investigate the effect of silver-containing dressings coverage after debridement on the repair of chronic refractory wounds from the aspects of wound infection and wound scars, in order to provide a reference for the treatment of chronic refractory wounds.

The article "Application Effect of Silver-Containing Dressings in the Repair of Chronic Refractory Wounds" was published in 2022. Journal: Evid Based Complement Alternat Med.

## 2. Materials and Methods

### 2.1. General Information

Eighty patients with chronic refractory wounds admitted from June 2019 to January 2022 were selected as the study subjects. The patients were randomly divided into a control group (*n* = 40) and an observation group (*n* = 40). The wound area of patients in the two groups was between 10 cm × 15 cm and 30 cm × 50 cm. All patients had slow granulation tissue growth, were not fresh, and had an ischemic pale appearance.

### 2.2. Standards

#### 2.2.1. Inclusion Criteria

The inclusion criteria were as follows: ① prolonged healing of ulcer wound for more than 2 weeks; ② no blood system disease; and ③ gave informed consent and was reviewed and approved by the Ethics Committee of the hospital.

#### 2.2.2. Exclusion Criteria

The exclusion criteria were as follows: ① anaerobic infection or wet gangrene; ② those who had used glucocorticoids and immunosuppressive agents and chemotherapeutic drugs; ③ wound caused by tumors; ④ confirmed allergy to silver preparations or dressings; and ⑤ poor compliance due to cognitive impairment, mental illness, etc.

### 2.3. Study Methods

All patients were given basic medical treatment such as diet control, nutritional improvement, smoking and alcohol deprivation, and application of antibiotics according to the bacterial examination of the wound.

The patients in the control group were treated with conventional dressing change methods: the wound surface was washed and disinfected, the necrotic tissue was removed, the drug was applied after hemostasis, the dressing change was regularly cleaned, an iodoform gauze or a gauze was placed to cover the wound surface according to the patient's wound surface; then, a sterile gauze or cotton pad was used to cover it. The dressing change time was determined according to the amount of exudate and secretion of the patient. The dressing change was started every day or every other day. When the wound surface was fresh or there was little secretion, the dressing change could be performed at an interval of 2-3 d.

The patients in the observation group were treated with silver-containing dressings for dressing change: first, the inactivated tissues in the wound surface and lacunae and the tissues prone to necrosis were completely removed, all lacunae were opened, and the wound skin was cleaned. An appropriately sized silver dressing (Biatain Alginate Ag, United Kingdom) was cut, the wound was sealed with a thin silver dressing pad on the wound, and the dressing needed to be replaced due to subsidence of the dressing. The wound was protected and compression of the wound was prevented from continuing, and the dressing was changed according to the wound condition for 1 day–3 days.

The article "Application Effect of Silver-Containing Dressings in the Repair of Chronic Refractory Wounds" was published in 2022. Journal: Evid Based Complement Alternat Med.

### 2.4. Observation Index

The observation indexes were as follows:

1. The degree of pain was compared between the two groups: the numerical rating scale (VAS) was used. The patients were counted as 0–10 points according to the degree of pain [9]. The patients scored the overall feelings of the two methods according to the dressing change period and assessed before treatment, 7 d, 14 d, and 1 month after treatment.
2. The dressing change and wound healing of the two groups were observed: the times of dressing change, granulation growth, wound formation, and healing time during treatment were statistically analyzed. Wound healing criteria: the wound area is less than 5% of the initial total area [10]. A transparent square paper of 0.25 cm × 0.25 cm was applied for measuring the wound area. Percentage of wound healing% = healing area/original wound area × 100%.
3. Wound scars in the two groups were observed: before treatment and after 1 month of treatment, the Vancouver Scar Scale (VSS) [11] was used to assess the thickness of the scar (0 indicates the same height as the surrounding normal skin, 1 indicates ≤2 mm higher than normal skin, 2 indicates 2 to 5 mm higher than normal skin, and 3 indicates >5 mm higher than normal skin), color (0 indicates that the scar color is similar to the skin of normal parts of the adjacent body, 1 indicates a slight pink color, 2 indicates a mixed color, and 3 indicates a darker color), softness (0 indicates normal, 1 indicates soft, 2 indicates flexible and bendable, 3 indicates hard, that is, inelastic and lumpy during hand pressure, 4 indicates that the tissue is cord-like, and 5 indicates contracture deformity), and vascularity (0 indicates that the scar color is similar to the normal parts of the body, 1 indicates that the pink local area is slightly higher, 2 indicates that the red local area is increased, and 3 indicates that the purple or dark red area is abundant) in four aspects, and the score indicates that the scar hyperplasia is more severe.
4. The wound infection of the two groups was observed: the wound was cultured for bacteria, and the results of bacterial culture were analyzed. The positive rate of bacterial culture before and after treatment was compared.

The article "Application Effect of Silver-Containing Dressings in the Repair of Chronic Refractory Wounds" was published in 2022. Journal: Evid Based Complement Alternat Med.

### 2.5. Statistical Methods

SPSS 22.0 software was applied for processing, and the measurement data of experimental data were analyzed using the mean ± standard deviation ($\bar{x}\pm s$), and enumeration data are expressed as (%) (metrological data). Pairwise comparisons were analyzed by *t*-test. Enumeration data were analyzed by the *χ*^2^ test. The test level is *α* = 0.05; *P* < 0.05 was considered statistically significant.

## 3. Results

### 3.1. Comparison of General Data between the Two Groups

There were no significant differences in gender, age, and wound area between the two groups (*P* > 0.05, Table 1).

### 3.2. Comparison of Pain Intensity between the Two Groups

There was no significant difference in the VAS score between the two groups before treatment (*P* > 0.05). The VAS score of the observation group decreased significantly after 7 days, 14 days, and 1 month of treatment, and the score was lower than that of the control group (Figure 1(a), 1(b)), and the differences were statistically significant (*P* < 0.05).

### 3.3. Comparison of Dressing Change and Wound Recovery between the Two Groups

The times of dressing change in the observation group were significantly less than that in the control group (Figure 2(a)). The granulation tissue growth time (Figure 2(b)), wound epithelialization time (Figure 2(c)), and wound healing time (Figure 2(d)) in the observation group were significantly higher than that in the control group, and the differences had a statistical significance (*P* < 0.05).

### 3.4. Comparison of Wound Scar between the Two Groups

There was no significant difference in wound scar before treatment between the two groups (*P* > 0.05). After treatment, the scores of wound scar thickness (Figure 3(a)), color (Figure 3(b)), softness (Figure 3(c)), and vascularity (Figure 3(d)) in the observation group were significantly reduced and the scores were significantly lower than those in the control group, and the differences had a statistical significance (*P* < 0.05).

### 3.5. Comparison of Wound Infection between the Two Groups

There was no significant difference in wound infection between the two groups before treatment (*P* > 0.05). After treatment, the positive rate of wound bacterial culture in the observation group was significantly lower than that in the control group (Figure 4), and the difference had a statistical significance (*P* < 0.05).

### 3.6. Analysis of a Typical Patient

The patient in the observation group, male, 28 year-old, was injured due to poor wound healing with an infection after right renal transplant resection (Figure 5(a)). After debridement, silver dressing was given to cover the day of treatment (Figure 5(b)). The granulation tissue grew well after 7 days of treatment, and there was no infection in the incision (Figure 5(c)). The dressing was continued for 46 days to heal (Figure 5(d)).

The article "Application Effect of Silver-Containing Dressings in the Repair of Chronic Refractory Wounds" was published in 2022. Journal: Evid Based Complement Alternat Med.

## 4. Discussion

Chronic refractory wounds have become one of the difficulties in the global health care field. With the in-depth understanding of the mechanism of chronic refractory wounds and the process of wound healing, a variety of theoretical systems have been proposed for chronic refractory wounds in clinic. The WBP theory focuses on the following four aspects of the wound that affect healing, namely, TIME: T (tissue nonviable) necrotic tissue, I (infection or inflammation) infection or inflammation, M (moisture imbalance) wet balance, and E (edge of wound) wound margin [12]. The TIME system was originally proposed by Schultz et al. [13], who focused on removing the bacterial, necrotic and cellular load affecting the wound surface, trying to maintain the wet balance of the wound surface, using various biological factors to actively create a relatively appropriate wound microenvironment, and accelerating wound healing or creating conditions for surgery. Supported by these scientific theories, the effect of silver ion dressing covering caused a hot debate.

Silver-containing dressings are composed of a 100% continuous nondeformable polyester fiber mesh hydrocolloid (sodium carboxymethylcellulose) and an antibacterial agent (silver ion complex). The mesh that is not easy to be deformed avoids the wound, can tolerate multiple mechanical stress effects, can be completely removed during dressing change, does not worry about dressing residues, and this dressing does not adhere to the wound and can significantly reduce pain [14, 15]. The dressing has a mesh which is not easy to deform, does not adhere to the wound, and can obviously relieve pain; and it can withstand mechanical stress for many times, which can be completely taken out during dressing change without leaving dressing [16–18]. In this study, after continuous treatment, the VAS score was significantly decreased, and the score in the observation group was lower than that in the control group. It is suggested that silver-containing dressings can not only continuously release highly active antibacterial silver ion but also has multiple effects such as absorbing exudate, promoting healing, no adhesion to wound surface, and preventing repeated injury caused by the next dressing change, indirectly reducing the pain level of dressing change for patients.

The article "Application Effect of Silver-Containing Dressings in the Repair of Chronic Refractory Wounds" was published in 2022. Journal: Evid Based Complement Alternat Med.

In this study, the times of dressing change in the observation group were significantly less than that in the control group, and the wound recovery of the patients in the observation group was significantly better than that in the control group. These results indicated that silver-containing dressings provided a moist healing environment for the wound surface and could promote granulation hyperplasia and epithelial tissue crawling. At the same time, our study found that the wound scar healing in the observation group was better than that in the control group. These results suggest that silver-containing dressings are beneficial to wound repair and accelerate the process of wound healing compared with common dressing. The reason is that silver-containing dressings are a clinical wound treatment material developed under the background of moist healing theory and wound negative pressure therapy theory, which can accelerate the healing of refractory wound and control the chronic infection of wound [19]. Once in contact with wound exudate, the hydrocolloid particle (CMC sodium carboxymethylcellulose) in the dressing swells after absorbing the exudate, forms a soft, cohesive hydrogel that allows it to absorb the wound exudate while locking it in place within the gel, avoiding the risk of exudate leakage as well as macerating the wound skin. Intrasite gel also creates a moist environment conducive to wound healing [20–22].

The results of this study showed that after treatment, the positive rate of wound bacterial culture in the observation group was significantly lower than that in the control group. Silver-containing dressings effectively eliminated susceptible bacteria, avoided the occurrence of clinical complications, and further ensured the cure rate of the disease. The reason why, silver sulfadiazine in silver dressings has a broad antibacterial spectrum and is active against both positive and negative bacteria, including molds and yeasts, especially *Staphylococcus aureus* and *Pseudomonas aeruginosa* (*Pseudomonas aeruginosa*) [23–25]. At the same time, the effective action time of the dressing is long, and after the silver ion-containing dressing loses its activity in the bacteria, the silver ion is freed from the bacteria and the bactericidal activity is repeated, with a longer antibacterial effect [26, 27]. Viruses and pathogenic bacteria will not produce drug resistance and drug resistance to them, so germs are not easy to produce variant varieties.

In summary, silver-containing dressings have a significant effect on the repair of chronic refractory wounds, which is conducive to reduce pain and scar hyperplasia, effectively promote the generation of granulation tissue and epithelial tissue and wound healing process, inhibit the growth of bacteria on the wound, and provide a reference for clinical treatment of chronic refractory wounds. The shortcoming of this study lies in the small included sample size and selective bias of the results. In the future, the sample size should be expanded to be confirmed by a more in-depth study.

The article "Application Effect of Silver-Containing Dressings in the Repair of Chronic Refractory Wounds" was published in 2022. Journal: Evid Based Complement Alternat Med.

## Figures and Tables

**Figure 1:** Comparison of pain intensity between the two groups. (a) Comparison of VAS scores between the two groups; (b) change trend of VAS score in two groups. ^*∗*^*P* < 0.05, compared with before treatment.

**Figure 2:** Comparison of dressing change and wound recovery between the two groups. (a) Dressing change; (b) the granulation tissue growth time; (c) wound epithelialization time; and (d) wound healing time. ^*∗*^*P* < 0.05, compared with before treatment.

**Figure 3:** Comparison of wound scar between the two groups. (a) Thickness; (b) color; (c) softness; and (d) vascularity. ^*∗*^*P* < 0.05, compared with before treatment.

**Figure 4:** Comparison of wound infection between the two groups. ^*∗*^*P* < 0.05, compared with before treatment.

**Figure 5:** Process of silver-containing dressings in the treatment of chronic refractory wound. (a) Before treatment; (b) on the day of treatment; (c) after 7 days of treatment; and (d) 46days to heal.

**Table 1:** Comparison of general data between the two groups.

Group	*N*	*Sex*	Age (years)	*Trauma site*		
		Male/Female		Thoracoabdominal	Extremities	Other

Control group	40	26/14	38.43 ±5.24	12	24	4
Observation group	40	27/13	39.05 ± 5.05	14	23	3
*t*/*χ*^2^ value		0.056	0.539	0.318		
*P* value		0.813	0.592	0.853		

Group	*N*	Wound area (cm^2^)	*Etiology*			
			Diabetic ulcer	Epilepsy	Radiation ulcer	Hot/Burn

Control group	40	29.45 ± 5.26	10	8	7	15
Observation group	40	30.92 ± 5.74	11	7	6	16
*t*/*χ*^2^ value		1.194	0.223			
*P* value		0.236	0.974			

## Data Availability

The data used and/or analyzed during the current study are available from the corresponding author on request.
